The article "Surgical Drill Guide for Insertion of an Infra-Acetabular Screw Based on an Anatomically Precontoured Plate System: A Cadaveric Study" was published in 2021. Journal: Biomed Res Int.

# Surgical Drill Guide for Insertion of an Infra-Acetabular Screw Based on an Anatomically Precontoured Plate System: A Cadaveric Study

**DOI:** 10.1155/2021/2321504

**Published:** 2021-07-26

**Authors:** Viola Freigang, Maximilian Gottsauner, Markus Rupp, Christian Pfeifer, Stephan Grechenig, Alexander Kerner, Volker Alt, Florian Baumann

**Affiliations:** ^1^Department of Trauma Surgery, Regensburg University Medical Center, Germany; ^2^Department of Cranio-Maxillofascial Surgery, Regensburg University Medical Center, Germany; ^3^Division of Macroscopic and Clinical Anatomy, Graz, Austria

## Abstract

**Purpose:**

Due to the anatomic structure of the pelvis, free-hand placement of screws in the acetabular fracture management can be difficult. Infra-acetabular screw fixation increases acetabular stability by distal fixation of the cup. Aim of this cadaveric study is to investigate if a plate-referenced drill guide can provide save placement of an infra-acetabular screw over a precontoured suprapectineal quadrilateral buttress plate (SQBP).

**Methods:**

We constructed a drill guide for an infra-acetabular screw based on the surface of an anatomically precontoured SQBP. A total of 12 adult cadaveric acetabular specimens were used for drill guide-assisted placement of the infra-acetabular screw. The drill guide contains a radiopaque spiral to allow longitudinal fine adjustment of the SQBP along the pelvic brim to assure correct position of the plate-drill-guide construct in relation to the Koehler's teardrop. After screw placement, we conducted a computed tomography (CT) scan of all specimens to assess the actual position of the screw in relation of the infra-acetabular corridor and the acetabular joint surface.

**Results:**

The position of the screw was within the infra-acetabular corridor in all cases. We did not see any intra-articular or intrapelvic screw penetration. The mean distance of the centerline of the screw to the medial border of the infra-acetabular corridor was 3.35 mm. The secure distance to the virtual surface of the femoral head to was 7.3 mm.

**Conclusions:**

A plate-referenced drill guide can provide safe placement of an infra-acetabular screw for treatment of acetabular fractures. Radiographic fine adjustment is necessary to access the optimal entry point.

## 1. Introduction

Due to the anatomic situation of the pelvis and acetabulum, management of an acetabular fracture is a technically demanding procedure. The close relationship to the iliac vessels and the complex construction of the acetabulum make it challenging to achieve reduction and fixation of the anterior and posterior acetabular column.

Demographic changes in industrial societies with overaging of the population have led to a shift in the typical fracture distribution. Large registry-based epidemiologic studies have demonstrated a rising number of acetabular fractures involving the anterior column over the last 20 years [1]. Limited bone mineral density is a frequent epiphenomenon in geriatric acetabular fractures and reduces fixation possibilities. A dissociation of the anterior column to the posterior column followed by a medialization of the quadrilateral surface has been identified as a risk factor for a secondary dislocation leading to a so called “central subluxation” of the femoral head [2–4]. As a consequence, a number of advancements concerning anterior approaches and fixation techniques have been made recently [2, 5–10]. Anatomically precontoured plate systems can provide enhanced reduction and fixation properties [10, 11]. Plate systems with a buttress to support the quadrilateral surface provide increased periacetabular stability [11–14].

The infra-acetabular screw following Letournel's [9, 12] concept of a periacetabular frame was reintroduced Culemann et al. in 2011 [13]. Marintshev et al. [14] proved increased stability with a screw inside the infra-acetabular corridor. Recently, a number of publications have investigated this bony corridor parallel to the quadrilateral surface centered in Koehler's teardrop [7, 15–17]. Since this corridor has a diameter of only few millimeters at level of the femoral head, the risk of an intraarticular screw placement for free-hand insertion is relatively high. A recently published radiomorphometric study revealed that the ideal entry point can be referenced to the tip of the iliopectineal eminence (IPE), and the drill angulation is remarkably constant in relation to the pelvic inlet plane (independent of age or gender) [15]. Anatomically precontoured suprapectineal plates show a convex bending reflecting the iliopectineal eminence. By matching the reference point (iliopectineal eminence) reflected by the convexity of the plate and the pelvic inlet plane (pectineal line) with the plate holes, a plate-referenced drill guide could ensure safe placement of an infra-acetabular screw.

The purpose of the study is to investigate if a plate-referenced drill guide can provide save placement of an infra-acetabular screw over a precontoured suprapectineal quadrilateral buttress plate (SQBP).

## 2. Materials and Methods

A total of 12 adult cadaveric acetabular specimens (6 pelvises) preserved by Thiel's method [18] were used in the presented study. The embalming method preserves color, consistency, and biomechanical properties of the musculoskeletal tissue. None of the pelvises showed signs of abnormity like skeletal dysplasia or prior bony injury of the acetabulum.

The specimens were dissected and stripped of the surrounding soft tissue. The hip joint capsule was dissected at level of the capsule-labral junction (Figure 1).

### 2.1. Drill Guide Construction

We matched a 3D-CAD model of the anatomically precontoured plate to a mean 3D surface model of 516 pelvises (SOMA, Stryker Orthopaedic Modeling and Analytics, Stryker Inc. Selzach, Switzerland). The shape of the surgical drill guide used in this study reflected the surface of the anatomically precontoured plate and had an optimal fit to the plate to assure a stable attachment of drill guide and plate. The drill guide was designed to contain the measurements determined in a recently published study on the ideal position of the infra-acetabular screw. Accordingly, the ideal entry point was 10.2 mm below and 10.4 mm medial to the highest point of the convexity of the plate reflecting the IPE. The angulation of the drill guide was in 10.4° to the axial plane and 71.4° to the sagittal plane of the pelvic inlet plane of the 3D model. The drill guide was constructed by additive manufacturing in a 3D-printing process.

### 2.2. Surgical Technique

For referencing of the drill guide position, we used a suprapectineal quadrilateral buttress plate (SQBP) (PRO pelvis supra-pectineal plate, Stryker Inc., Selzach, Switzerland). The plate was placed aiming for an optimal fit of the anatomical precontoured shape and fixed starting with a parasymphysial screw and pressing the plate laterally to achieve an adequate fit on the pelvic brim to assure alignment with the pelvic inlet plane (Figure 1). Preliminary tests showed that this surgical routine-based proceeding missed required accuracy to access the optimal entry point of the infra-acetabular corridor. Fluoroscopic images revealed that there is somewhat longitudinal displaceability of the SQBP along the pelvic brim in direction of the linea terminalis.

Therefore, we added a radiopaque spiral to the drill guide to assure the correct position of the plate-drill-guide construct in relation to Koehler's teardrop (Figure 2). A fluoroscopic image in a combined obturator oblique outlet view was taken to assure overlap of the radiopaque spiral and Koehler's teardrop. Then, the plate was fixed by iliacal and pubic screws according to the surgical technique provided by the plate manufacturer (https://otaonline.org/industry-partners/stryker/multimedia/16879679/pro-pelvis-suprapectineal-plate-placement). After secure placement of the plate, we attached the drill guide to the plate and inserted another screw in the medial part of the plate (against the quadrilateral buttress) to secure the drill guide position and to avoid mediolateral tilting of the plate. After that, a 2.5 mm hole was drilled through the drill sleeve. The drill contained a depth measuring scale which was used to determine the length of the screw.

After insertion of the screw, the plate and the screws through the plate were removed leaving only the infra-acetabular screw in place to reduce material artifacts of the computed tomography (CT) scan. Since the screw does not go through a plate hole, the plate could be removed without the risk of malplacement when reinserting the infra-acetabular screw.

### 2.3. Radiographic Measurement

After drill guide-assisted placement of the infra-acetabular screw, we conducted a CT scan of all specimens to assess the actual position of the screw in relation of the infra-acetabular corridor and the acetabular joint surface. The position of the screw was measured using a picture archiving and communication system (PACS) software (Osirix 5.9, Pixmeo SARL, Bern, Switzerland). The infra-acetabular corridor was evaluated in a CT reconstruction plane centered at level of the infra-acetabular corridor with an inlet angulation of 25° according to Kanezaki and Miyazaki [16]. We characterized the infra-acetabular corridor by the diameter of the corridor perpendicular to the center of the femoral head center (IAD: infra-acetabular diameter), the distance of the center of the corridor to the virtual femoral head cartilage surface (CCD: center cartilage distance), and the length of the infra-acetabular corridor (IACL: infra-acetabular corridor length) measured by the screw length.

The measurement of the relation of the femoral head and the infra-acetabular screw was identified by generating a multiplanar reformation (MPR) centered through the core of the screw and the center of the femoral head according to Egli et al. [10] (Figure 3).

The distance of the center of the screw to the medial wall of the infra-acetabular corridor at level of the center of the femoral head (SCD: screw-corridor distance): To measure the distance of the center of the screw to the virtual cartilage surface of the femoral head (SFHD: screw femoral head distance), we drew a virtual circle along the chondral border of the acetabulum to simulate the cartilage border of the head. All measurement results were recorded in mm.

The cadaveric specimens were donated to the university anatomy program. Donors gave their informed written consent for the donation and anatomical dissection during lifetime. No further prehumous data like medical records were used in this study. Therefore, there was no necessity for an approval by an ethics committee.

### 2.4. Statistical Analysis

Statistical analysis was performed using the software package SPSS (Version 25, SPSS Inc, Chicago, Illinois). Since there is no previous data, this preliminary study was designed as an exploratory pilot study without any *a* priori sample size calculation based on a primary endpoint. Based on the low variance of values in the previous radiomorphometric study and based on other experimental studies, a sample size of 12 specimens was considered feasible and expected to have enough power [16, 19]. Unless otherwise stated, descriptive data are given as mean ± standard deviation.

## 3. Results

The position of the screw was within the infra-acetabular corridor in all cases. We did not see any intra-articular or intrapelvic screw penetration.  Table 1 shows measurement results recorded in 12 cadaveric acetabula. The mean diameter of the virtual femoral head was 45.1 mm (±2.6). The infra-acetabular corridor had a mean width (IAD) of 6.93 mm (±0.81) at level of the femoral head center. The mean distance of the middle of the corridor to the virtual cartilage surface of the femoral head (CCD) was 7.53 mm (±1.42).

The mean corridor length measured at level of the screw (IACL) was 88.4 mm (±7.4). The mean distance of the core of the screw to the medial wall of the infra-acetabular corridor (SCD) was 3.36 mm (±0.83). The secure distance between screw and the virtual femoral head cartilage surface (SFHD) was 7.30 mm (±1.71).

## 4. Discussion

This feasibility study demonstrated that a save placement of an infra-acetabular screw is possible by a plate-referenced drill guide over a precontoured SQBP. The entry point and angulation of the drill guide enabled save advancement of the drill directly into the infra-acetabular corridor. However, radiographic fine adjustment of the plate-drill-guide construct is indispensable to assure correct placement of the plate along the pelvic brim.

The secure distance between screw and the virtual femoral head cartilage surface was 7.30 mm (SFHD).

Demographic changes lead to an overaging of industrial societies and a rising number of geriatric fractures with a typical fracture pattern due to reduced bone quality in elderly [1, 3, 20, 21]. Geriatric acetabular fractures typically involve the anterior column of the acetabulum. In the past, fractures involving the posterior wall or posterior column were much more frequent. The posterior Kocher/Langenbeck approach was the standard approach in treatment of fractures of the acetabulum [12, 22]. Within the past two decades, more and more geriatric fractures occur so that anterior approaches are used most frequent today [1, 8]. This trend initiated further advancement of anterior approaches and operative techniques via anterior approaches [2, 4, 14, 23–27]. In 1993, Letournel was the first to describe a screw position through the acetabular fossa parallel to quadrilateral surface to increase intrinsic acetabular stability by a periacetabular frame construct [9].

Based on the quadrilateral screw described by Letournel [9], Culemann et al. [13] published a modified quadrilateral screw inserted more inferior in the region of Koehler's teardrop in 2011. This so-called “infra-acetabular” screw was intended to fix the anterior to the posterior column and to minimize the risk of intraarticular penetration of the screw. A biomechanical study by Gras et al. [24] found that an infra-acetabular screw significantly increases the stability of the acetabular fixation construct compared to a standard plate fixation. Standard implant size in management of acetabular fractures is a screw diameter of 3.5 mm requiring a drill hole for the infra-acetabular screw of 2.5 mm. Drill guide-based drilling might provide enough accuracy for a secure placement of screws even in a narrow bony canal like the infra-acetabular corridor.

In cases of reduced bone quality, a simple fall can cause a fracture of the anteromedial acetabulum or the quadrilateral surface by load transmission through the major trochanter [28]. A lack of support of the quadrilateral surface has been identified as a risk factor for a secondary dislocation leading to a so-called “central sub-luxation” of the femoral head [4, 20, 21, 24, 29]. In recent years, different concepts were introduced to increase medial support of the quadrilateral surface to prevent this complication [2, 4, 13, 14, 23, 24, 27, 28, 30]. Besides new plate designs like the SQBP and a screw placement close to the joint surface, the infra-acetabular screw has increasingly attracted attention the discussion on advancements in acetabular fracture management [10, 16, 31].

Intra-articular screw penetration can cause a cartilage damage of the femoral head. We did not see any intra-articular screw position. The CT measurements revealed a secure distance of the screw to the femoral cartilage surface of 7.30 mm (SFHD). The diameter of the infra-acetabular corridor at level of the femoral head center was 6.72 mm.

Recently, a large biomorphometric CT-based study identified a viable infra-acetabular corridor with a diameter over 5 mm in 93% of specimens [7]. Due to variance of the pelvic morphology, referencing of the entry point to anatomic landmarks like the pubic symphysis is not accurate enough for clinical practice. Recently, a radiomorphometric study referenced the ideal entry point of the infra-acetabular screw 1 cm caudal and medial to the IPE in an angulation of 10° in the axial plane and 70° in the sagittal plane.

Instead of referencing the drill guide to the bony surface that might vary between each patient, the drill guide was referenced to a SQBP with a standardized surface. Using the plate as a reference, the interface between drill guide and plate allows an accurate fit without any deviation of the drill. Altering the level of patient-specific adjustment to the interface between plate and bone surface enlarges contact surface minimizing the risk of discrepancy of drilling direction in regard of the infra-acetabular corridor. In addition, conducting the drill process after insertion of the plate allows more room of action for the surgeon. The window of the intrapelvic approach provides a good overview and access to the anterior column and the quadrilateral surface. However, it can be difficult to manipulate with bulky instruments in the depth of the pelvis. Assembling the plate drill guide like a modular construct in situ might have an advantage over a large monobloc drill guide detecting the bone surface directly. The plate is constructed of annealed stainless steel which allows bending of the plate according to the bony surface. This implies the risk of mismatch of the drill guide and the plate when adaption by bending. His bending can also occur unintentionally by screw insertion and compression of the plate bone interface This has to be taken into account as a potential cause of mismatch of the plate-drill-guide interface and consequentially misguidance of the drill. However, most of the deflection of the plate takes place on the edges of the plate and the triangular shape of the plate at level of the drill guide prevents bending at this area. We did not observe any deflection of the plate at level of the plate-drill-guide interface leading to a mismatch or deviation of the drill. There is also a trend towards personalized medicine. Several pilot studies have proven advantages of preoperative 3D model-based plate bending for acetabulum fractures [27, 32, 33]. Although this procedure is time consuming and costly, this may become the standard of care making a bending of the plate evitable.

There is an ongoing debate about “safe zones” and “un-safe zones” in acetabular fracture management [34]. The entry point of the infra-acetabular screw is located in an unsafe zone. Even with the knowledge of the ideal entry point, free-hand insertion implicates the risk of an intra-articular screw position. Therefore, a drill guide-based insertion could be rewarding to replicate the ideal drill hole for an infra-acetabular screw. The plate-referenced drill guide used in this study allowed save placement of an infra-acetabular screw over a precontoured SQBP in all cases. Further studies are necessary for clinical implementation.

This study has some limitations. We manufactured the drill guide based on the SQBP that is adapted to a mean pelvic model based on 516 pelvic 3D CT scans of healthy subjects. This construction might not be suitable for patients with extreme skeletal dysplasia or degeneration of the hip joint. However, the pelvises used in this cadaveric study were of geriatric subjects with degenerative changes with a deep acetabular fossa narrowing the infra-acetabular canal. Even in these cases, we did not record any intra-articular screw penetration. Another limitation is that the drill guide was applied in not fractured acetabular cadavers. Incongruence of the infra-acetabular corridor due to insufficient reduction in a fracture situation can lead to occlusion of the designated screw canal or discrepancy of the reference at level of the quadrilateral surface. The limited number of cadavers that we used in this study reduces generalizability. Intention of this preliminary pilot study was to prove the principle of SQBP-based drill guide screw placement and to gain practical experience.

Detection of longitudinal displaceability of the SQBP along the pelvic brim in direction of the linea terminalis was one of the major findings that can only be detected in practical application. Although we did not observe any deformation of the plate, this could lead to a mismatch of the plate and drill guide leading to deviation of the drill.

Further studies are necessary to proof reliability in a large number of cases and in clinical application.

## 5. Conclusion

A plate-referenced drill guide can provide safe placement of an infra-acetabular screw for treatment of acetabular fractures. Radiographic fine adjustment is necessary to access the optimal entry. The secure distance between screw and the virtual femoral head cartilage surface was 7.30 mm (SFHD). Further studies are needed to proof reliability in clinics.

## Figures and Tables

**Figure 1:** Fixation of the plate and drill guide construct to a left acetabulum (a) and image showing the infra-acetabular screw (white arrow) after removal of the plate (b).

**Figure 2:** Fluoroscopy image for fine adjustment of the plate position (a) and an image showing the relation of Koehler's teardrop (center of the metal ring) and the drill guide (b) in a combined inlet oblique view along the infra-acetabular canal. Drill guide with a radiographic marker on a left acetabulum (c).

**Figure 3:** Screenshot illustrating software-based measurements of the CT-based MPR.

**Table 1:** Results of the computed tomography-based multiplanar reformation measurements given in mm.

Specimen No.	Infra-acetabular diameter (IAD)	Center cartillage distance (CCD)	Infra-acetabular corridor length (IACL)	Screw corridor distance (SCD)	Screw femoral head distance (SFHD)	Femoral head diameter (FHD)
1L	7.90	6.96	79.6	3.62	7.01	42.7
1R	8.06	7.12	80.7	3.24	6.52	42.3
2R	6.56	8.30	84.9	3.13	7.74	43.4
2L	6.68	8.34	81.1	2.41	6.70	43.4
3R	6.53	7.90	85.7	3.14	7.68	49.6
3L	6.89	7.31	99.9	2.72	6.99	50.1
4R	5.83	6.36	99.8	2.98	6.72	43.0
4L	7.08	7.39	85.9	3.29	6.80	42.8
5R	6.19	7.61	98.5	3.14	7.17	46.4
5L	5.87	4.15	92.0	2.66	3.73	46.2
6R	8.12	9.30	85.9	4.95	9.98	45,2
6L	7.44	9.57	86.9	5.05	10.50	45.8
Mean	6.72	7.62	90.1	3.35	7.40	45.6
Range	0.71	1.54	7.0	0.91	1.87	2.6
Min	5.83	4.15	81.1	2.41	3.73	2.6
Max	8.12	9.57	99.9	5.05	10.50	50.1

## Data Availability

Please contact the author for data requests.

## Abbreviations

CCD: Center cartilage distance
CT: Computer tomography
IACL: Infra-acetabular corridor length
IAD: Infra-acetabular diameter
IPE: Iliopubic/Iliopectineal eminence
MPR: Multiplanar reformation
PACS: Picture archiving and communication software
SCD: Screw corridor distance
SFHD: Screw femoral head distance
SQBP: Suprapectineal quadrilateral buttress plate.
